# Knockdown of small nucleolar RNA host gene 10 (SNHG10) alleviates the injury of human neuroblastoma cells via the miR-1277-5p/insulin substrate receptor 2 axis

**DOI:** 10.1080/21655979.2021.2012623

**Published:** 2021-12-30

**Authors:** Zhaoming Sun, Lixiang Song, Jiazhen Li

**Affiliations:** Department of Neurology, Yantai Yuhuangding Hospital Affiliated to Qingdao University, Yantai, Shandong, China

**Keywords:** SNHG10, miR-1277-5p, IRS2, Parkinson’s disease

## Abstract

Parkinson’s disease is a common neurodegenerative disease with a complex physio-pathology. So far, there is no effective medical strategies to prevent the progression of Parkinson’s disease. Understanding the mechanisms underlying the progression of Parkinson’s disease could provide insights into the formulation of novel preventative or treatment strategies. Small nucleolar RNA host gene 10 (SNHG10) is a lncRNA which has been implicated in the development of many cancers. However, its potential role in Parkinson’s disease remains unknown. In this study, we found that SNHG10 was upregulated while miR-1277-5p was downregulated in the Parkinson’s disease cell model of 1-Methyl-4-phenyl-pyridine ion (MPP+) induced SH-SY5Y cells. We further revealed that SNHG10 sponged miR-1277-5p to negatively regulate its expression, and miR-1277-5p could bind to the 3′UTR of insulin substrate receptor 2 (IRS2) mRNA to suppress its expression. These data suggest that SNHG10 regulates IRS2 through interacting with miR-1277-5p in the cell model of Parkinson’s disease. Through a series of molecular experiments and functional assays, we demonstrated that downregulating SNHG10 in the cell model of Parkinson’s disease attenuated the cell injury by reducing the expression of IRS2. Meanwhile, inhibiting miR-1277-5p or overexpressing IRS2 could partially reverse the effect of SNHG10 knockdown. In summary, our data indicate that knockdown of SNHG10 mitigates MPP^+^ induced damage in SH-SY5Y cells via the miR-1277-5p/IRS2 axis.

## Introduction

Parkinson’s disease is the second common neurodegenerative disease in the central nervous system and approximately 6 million individuals are diagnosed with Parkinson’s disease yearly [1]. Parkinson’s disease is characterized by the loss of dopaminergic neurons in the nigrostriatal system, accompanied by the motor and nonmotor symptoms. Current medicines may delay the symptoms but fail to prevent the disease progression. Previous studies suggest that Parkinson’s disease is a heterogeneous disorder in terms of etiologies, clinical symptoms, and diagnosis [2]. Many factors, including environment, age, and genetics, can promote the loss of dopaminergic neurons [3,4]. The precise cause of Parkinson’s disease remains unknown. Understanding the mechanisms underlying the progression of Parkinson’s disease could provide insights into the formulation of novel preventative or treatment strategies.

Long non-coding RNAs (lncRNAs) are non-coding RNAs with more than 200 nucleotides [5]. Accumulating evidence reveals that lncRNAs are implicated in a variety of human diseases, including Parkinson’s disease [5–7]. Recent studies have demonstrated that lncRNA SNHG10 plays important roles in various tumors [8–13]. However, its role in Parkinson’s disease is unclear. In many scenarios, lncRNAs act as a sponge of microRNAs (miRNAs) to regulate downstream target mRNA [14,15]. miRNAs are non-coding RNAs with about 22 nucleotides [16], which play critical roles in regulating gene translation [16].

Recently, miR-1277-5p has been reported as a low-expression miRNA in the cell model of Parkinson’s disease [17]. Using Starbase database for lncRNA-miRNA interaction prediction, we found that SNHG10 could potentially target miR-1277-5p. We also find that Insulin substrate receptor 2 (IRS2), which is a cytoplasmic adaptor protein of insulin signaling pathway [18], is a target of miR-1277-5p. Since IRS2 shows a highly expression in the cell model of Parkinson’s disease [19], we therefore hypothesized that the interactions among SNHG10, miR-1277-50, and IRS2 play important roles in the Parkinson’s disease. Through a series of molecular experiments and functional assays, we demonstrated that downregulating SNHG10 in the cell model of Parkinson’s disease attenuated the cell injury by reducing the expression of IRS2. Meanwhile, inhibiting miR-1277-5p or overexpressing IRS2 could partially reverse the effect of SNHG10 knockdown. In summary, our data indicate that knockdown of SNHG10 mitigates MPP+ induced damage in SH-SY5Y cells via the miR-1277-5p/IRS2 axis.

## Materials and methods

### Cell culture and MPP+ treatment

Human neuroblastoma cell line SH-SY5Y (American Tissue Culture Colection) were cultured in Dulbecco’s Modified Eagle Media: Nutrient Mixture F-12 (DMEM/F12), supplemented with 10% fetal bovine serum (FBS, Gibco, USA) and 1% penicillin/streptomycin (Gibco, USA) in a humidified incubator at 37°C, 5% CO_2_. 5 mM MPP^+^ (1-Methyl-4-phenylpyridinium iodide, D048-1 G. Sigma, USA) was added into cell culture for 18 h to establish the cell model of Parkinson’s disease.

### qRT-PCR (quantitative real-time PCR)

Trizol reagent (15,596,026, Thermo Fisher Scientific) was used to extract RNA from cells according to the manufacturer’s instructions. 1 μg of total RNA was used for reverse-transcription into cDNA using RevertAid First Strand cDNA Synthesis Kit (K1622, Thermo Fisher Scientific). Diluted cDNA was analyzed in a 7500 Real Time PCR System (Applied Biosystems/Life Technologies, Carlsbad, CA, USA) using SYBR Select Master Mix (Takara, Dalian, China). The PCR cycling condition used: 95°C 5 mins, 40 cycles of 95°C 30 sec, 60 ℃ 30 sec and 72 ℃ 60 sec. The 2^–∆∆Ct^ method was used to analyze the relative expression level and Glyceraldehyde-3-phosphate dehydrogenase (GAPDH) and U6 were used as the internal reference genes. All primer sequences were synthesized and purchased from Shanghai Sangon Biotechnology Co., Ltd. (Shanghai, China): SNHG10 forward: CCAGCTTAGATTCATTGATTCC, SNHG10 reverse: TTAAGTGCACCAGATGCTG; GAPDH forward: GAACGGGAAGCTCACTGG, GAPDH reverse: GCCTGCTTCACCACCTTCT; miR-1277-5p primary sequence: AAAUAUAUAUAUAUAUGUACGUAU; U6 forward: CTCGCTTCGGCAGCACA, U6 reverse: AACGCTTCACGAATTTGCGT.

### Cell transfection

miR-1277-5p mimic, miR-1277-5p inhibitor, miR-NC, control siRNA, SNHG10 siRNA and vector expressing IRS2 were purchased from Guangzhou RiboBio (Guangzhou, China). Transfections of above molecules into the cells were performed by Lipofectamine 3000 (Invitrogen, Carlsbad, CA) following the manufacturer’s protocol. 4 µg plasmid and 200 nM of miR-345-3p mimic or the NC were used for transfecting cells in 6 well plate with 80% confluency. 48 h after transfection, cells were harvested for further experiments.

### Western blot

Total protein was extracted from cells using RIPA lysis buffer containing protease inhibitor cocktail (Thermo Fisher Scientific, Waltham, MA, USA). Cells suspended in RIPA buffer were lysed on ice for 10 mins and lysed cells were centrifuged at 14,000 rpm for 10 mins. The supernatant containing total protein lysate was quantified by a BCA Protein assay kit (Beyotime Biotechnology P0009; Shanghai, China). 20 µg of protein was loaded into 12% sodium dodecyl sulfate salt-polyacrylamide gel electrophoresis (SDS-PAGE) gel and transferred onto a polyvinylidene fluoride (PVDF) membrane. After blocking with 5% skimmed milk the membrane was incubated with primary antibody IRS2 (1:5000, Abcam) overnight at 4°C. The membrane was washed 3 times with TBST for 5 minutes each. After wash, the membrane was further incubated with HRP-linked secondary antibody (1:2500; Cell Signaling Technologies, MA, USA) at room temperature for 1 hour. Then the membrane was washed 4 times with TBST and the protein bands were visualized using an Electro-Chemi-Luminescence kit (Santa Cruz, TX, USA) and photographed on a gel imager system (Bio-Rad, Hercules, CA, United States). The densitometry analysis was performed with Image J software (Bethesda, MD, USA) [20].

### Enzyme Linked Immune Sorbent Assay (ELISA)

The levels of tumor necrosis factor α (TNF-α), interleukin 1β (IL-1β), IL-6, reactive oxygen species (ROS), malondialdehyde (MDA), and superoxide dismutase (SOD) were measured by ELISA using 100 µL cell culture supernatant. The ELISA kits were used from ABIOCENTER (Beijing, China). The procedures were performed according to the instructions of manufacturer.

### Cell Counting Kit 8 (CCK-8)

Cells were seeded in to a 96-well plate at a density of 1500 cell/well and cultured in a humidified cell culture incubator for 0, 24, 48, and 72 hours, respectively. Subsequently, 10 μl CCK8 reaction solution (Beyotime, Shanghai, China) was added to the cell culture at indicated time point and incubated for 1 hour in a humidified cell culture incubator. The light absorption value (OD value) in each condition was captured at 450 nm wave length on a Synergy H1 microplate reader (Winooski, Vermont, USA).

### Apoptosis detection by flow cytometry

The detection of cell apoptosis was performed using the FITC Annexin V Apoptosis Detection Kit (BD Biosciences, CA, USA) according to the manufacturer’s instructions. Briefly, cells with different treatments were trypsinized and washed twice with 1x PBS, and resuspended in the 1 ml staining solution containing 5 μL Annexin V-FITC and 5 μL PI. The cells were incubated for 30 min in the dark and washed twice with 1x PBS. The percentage of apoptotic cells was detected by BD FACS CantoTM II Flow Cytometer (BD Biosciences).

### Luciferase reporter assay

The potential interactions of SNHG10 and miR-1277-5p and miR-1277-5p and IRS2 were examined by the luciferase reporter assay in SH-SY5Y cells. The wild-type SNHG10 sequence and IRS2 3ʹUTR sequence containing miR-1277-5p complementary sites, or the mutated sequences were cloned into PmirGLO vector expressing firefly luciferase (Promega, USA). The reporter plasmid and Renilla luciferase (hRlucneo) control plasmid were co-transfected into cells with either miR-1277-5p mimic or miR-NC in a 12-well plate (1 × 10^5^ cells/well) using Lipofectamine 3000 reagent according to the manufacturer’s instructions (Invitrogen, L3000001). The relative luciferase activities were measured using Dual-Luciferase Reporter Assay Kit (Promega, E1910) on a luminescence microplate reader (Infinite 200 PRO; Tecan) 48 h after transfection. The relative firefly luciferase activity in the reporter plasmid was normalized to that of Renilla luciferase (hRlucneo) control plasmid [21].

### RNA pull-down

The biotinylated SNHG10 oligonucleotide probe or control probe (Genechem, China) were transfected into SH-SY5Y cells. 24 h after transfection, cell lysates were collected by IP lysis buffer (Beyotime, P0013). 10% of the lysates was saved as the input. The remaining lysates were incubated 100 µl M-280 streptavidin magnetic beads (Sigma-Aldrich, 11205D) at 4°C overnight. A magnetic bar was used to pull down the magnetic beads and associated nucleic acids, then the samples were washed 4 times with high salt wash buffer. Both the input and the elutes from the pull-down experiments were purified with Trizol reagent (15,596,026, Thermo Fisher Scientific) according to the manufacturer’s protocol [22]. Reverse transcription and quantitative RT-PCR analysis were performed as described in qRT-PCR (quantitative real-time PCR) section.

### Statistical analysis

Data are expressed as mean ± SD. We used a two-tailed unpaired Students’ t test to determine differences between two groups. One-way analysis of variance (ANOVA) was used to compare the differences among multi-groups, with Tukey’s post hoc test for pairwise comparison. Comparisons of data at multiple time points were examined using two-way ANOVA. All statistical analyses were performed using the Statistical Package for the Social Sciences version 23.0. p < 0.05 was considered statistically significant.

## Results

In this study, we found that SNHG10 could target miR-1277-5p, and miR-1277-5p in turns regulates the expression of Insulin substrate receptor 2 (IRS2). Since IRS2 shows a high-level expression in the cell model of Parkinson’s disease [19], we further investigated the functional interactions among SNHG10, miR-1277-50, and IRS2 in the cell model of Parkinson’s disease. We demonstrated that downregulating SNHG10 in the cell model of Parkinson’s disease attenuated the cell injury by reducing the expression of IRS2. In addition, miR-1277-5p inhibition or IRS2 overexpression could partially reverse the effect of SNHG10 knockdown. Our data collectively indicate that knockdown of SNHG10 mitigates MPP+ induced damage in SH-SY5Y cells via the miR-1277-5p/IRS2 axis.

### Downregulating SNHG10 attenuated the cell injury in the cell model of Parkinson’s disease

In a Parkinson’s disease model of MPP+ induced SH-SY5Y cells, we first examined the expression level and the functional role of SNHG10 and miR-1277-5p. qRT-PCR analysis revealed that the expression level of SNHG10 was increased while the expression of miR-1277-5p was decreased after MPP+ treatment (Figure 1). We next transfected cells with a siRNA targeting SNHG10, which could efficiently downregulate the expression of SNHG10 in the cell model of Parkinson’s disease (Figure 2a). CCK-8 proliferation assay and flow cytometry-based apoptotic assay demonstrated that the downregulation of SNHG10 promoted cell proliferation and attenuated apoptosis in the cell model of Parkinson’s disease (Figure 2b). We further performed ELISA and found that MPP+ treatment increased the level of pro-inflammatory cytokines, including TNF-α, IL-1β, and IL-6, while downregulating SNHG10 decreased their levels (Figure 2d). Meanwhile, cellular oxidative stress (ROS and MDA) elicited by MPP+ was also attenuated by SNHG10 knockdown, which was accompanied by the increased level of antioxidant enzyme SOD (Figure 2g-i). Together, these data indicate that downregulating SNHG10 attenuated the cell injury of SH-SY5Y cells in the cell model of Parkinson’s disease.

**Figure 1.** **In the MPP^+^-induced SH-SY5Y cells, the expression level of SNHG10 is increased while miR-1277-5p expression is reduced**. (a) qRT-PCR analysis of the expression level of SNHG10 in the MPP^+^-induced SH-SY5Y cells (p < 0.001). (b) qRT-PCR analysis of the expression level of miR-1277-5p in the MPP^+^-induced SH-SY5Y cells (p < 0.01). Data are the summary of 3 independent experiments.

**Figure 2.** **Downregulating SNHG10 attenuates cellular stresses in MPP^+^ induced-SH-SY5Y cells**. (a) qRT-PCR analysis of SNHG10 expression level in SNHG10 silenced cells (p < 0.001). (b) CCK-8 proliferation assay in MPP+ induced SH-SY5Y cells with or without SNHG10 silencing. (c) Flow-cytometry based apoptosis detection in MPP+ induced SH-SY5Y cells with or without SNHG10 silencing. (d-i) ELISA was performed to detect (d) TNF-α, (e) IL-1β, (f) IL-6, (g) ROS level, (h) MDA and (i) SOD in MPP+ induced SH-SY5Y cells with or without SNHG10 silencing. Data are the summary of 3 independent experiments. *p < 0.05, **p < 0.01, ***p < 0.001.

### SNHG10 targets miR-1277-5p and downregulating miR-1277-5p partially reverses the effect of SNHG10 knockdown in the cell model of Parkinson’s disease

Next, we attempted to find the downstream target of SNHG10 in the cell model of Parkinson’s disease. Via the Starbase database, we found that the 3ʹUTR region of SNHG10 contained a potential miR-1277-5p binding site (Figure 3a). To verify their functional interaction, we performed dual-luciferase reporter assay using both WT reporter or MUT reporter containing mutated binding site. The presence of miR-1277-5p mimic suppressed the luciferase activity of ET reporter, but no effect was observed in MUT reporter (Figure 3b). In addition, RNA pull-down experiment confirmed that in the SH-SY5Y cells, SNHG10 probe can significantly enriched miR-1277-5p as compared to the control (NC) probe (Figure 3c). When SNHG10 was silenced by siRNA, the expression level of miR-1277-5p was significantly increased (Figure 3d). These data collectively showed that SNHG10 targets miR-1277-5p and negatively regulates its expression in the SH-SY5Y cells.

**Figure 3.** **miR-1277-5p is a target of SNHG10**. (a) Using Starbase database, miR-1277-5p was found as a target of SNHG10. (b) Dual luciferase activity assay using wildtype (WT) or mutated binding site (MUT) reporter, in the presence or absence of miR-1277-5p mimic. (c) RNA pull-down assay using control probe (NC group) or SNHG10 probe in SH-SY5Y cells. The precipitated miR-1277-5p level was quantified by qRT-PCR and normalized to the input. (d) qRT-PCR analysis of miR-1277-5p after SNHG10 knockdown by si-SNHG10 group. Data are the summary of 3 independent experiments. ***p < 0.001.

We next sought to validate whether miR-1277-5p mediates the functional role of SNHG10. In the SH-SY5Y cells, we first confirmed that miR-1277-5p inhibitor significantly decreased the expression of miR-1277-5p (Figure 4a). In the cell model of Parkinson’s disease induced by MPP+, we performed CCK-8 and apoptosis assay after SNHG10 knockdown in the presence of miR-1277-5p inhibitor. We found that inhibiting miR-1277-5p suppressed the cell proliferation and increased apoptosis after downregulating SNHG10 (Figure 4b and c). ELISA measurement further demonstrated that downregulating miR-1277-5p partially increased the inflammatory cytokine levels and the cellular oxidative stress level after SNHG10 knockdown (Figure 4d). In summary, these data suggest that miR-1277-5p mediates the functional roles of SNHG10 in the cell model of Parkinson’s disease.

**Figure 4.** **Downregulating miR-1277-5p partially reverses the effects of SNHG10 silencing**. (a) In the SH-SY5Y cells, compared with the control (NC inhibitor group), miR-1277-5p inhibitor significantly decreased the level of miR-1277-5p. (b) CCK-8 proliferation assay in MPP+ induced SH-SY5Y cells with or without SNHG10 silencing and miR-1277-5p inhibitor. (c) Flow-cytometry based apoptosis detection in MPP+ induced SH-SY5Y cells with or without SNHG10 silencing and miR-1277-5p inhibitor. (d-i) ELISA was performed to detect (d) TNF-α, (e) IL-1β, (f) IL-6, (g) ROS level, (h) MDA and (i) SOD in MPP+ induced SH-SY5Y cells with or without SNHG10 silencing and miR-1277-5p inhibitor. Data are the summary of 3 independent experiments. *p < 0.05, **p < 0.01, ***p < 0.001.

### SNHG10 regulates IRS2 expression by sponging miR-1277-5p in SH-SY5Y cells

We next determined the target of miR-1277-5p in SH-SY5Y cells. Using the microRNA target prediction online tool (Starbase database), miR-1277-5p appeared to bind to the 3′UTR of IRS2 region (Figure 5a). Based on the dual luciferase report assay, we found that miR-1277-5p mimic inhibited the activity of WT reporter containing IRS2/miR-1277-5p binding site, while no effect was observed in the MUT reporter (Figure 5a). In SH-SY5Y cells, upregulating miR-1277-5p by transfecting with miR-1277-5p significantly decreased the protein level of IRS2 (Figure 5b). These data strongly indicate that miR-1277-5p regulates the expression of IRS2.

**Figure 5.** **SNHG10 regulates the expression of IRS2 by sponging miR-1277-5p**. (a) Based on Starbase database, miR-1277-5p binds to the 3′UTR of IRS2 region. In the SH-SY5Y cells, dual luciferase activity assay using wildtype (WT) or mutated binding site (MUT) reporter, in the presence or absence of miR-1277-5p mimic. (b) Western blot analysis of IRS2 protein level in SH-SY5Y cells transfected with miR-NC and miR-1277-5p mimic. (c) Western blot analysis of IRS2 protein levels in MPP+ induced cells with SNHG10 silencing and miR-1277-5p inhibitor. (d) qRT-PCR analysis of the mRNA level of IRS2 in MPP+ induced cells. (e) Western blot analysis of IRS2 protein level in MPP+ induced cells. Data are the summary of 3 independent experiments. **p < 0.01, ***p < 0.001.

To determine whether SNHG10 could regulate IRS2 expression through miR-1277-5p, we silenced SNHG10 in MPP+ induced SH-SY5Y cells, with or without miR-1277-5p inhibitor. Silencing SNHG10 significantly decreased the protein expression of IRS2. The presence of miR-1277-5p inhibitor significantly reversed the effect of SNHG10 silencing by increasing IRS2 level (Figure 5c). In addition, in the cell model of Parkinson’s disease, the mRNA and protein levels of IRS2 were significantly increased (Figure 5d and e). Therefore, we conclude that SNHG10 regulates the expression of IRS2 by sponging miR-1277-5p in SH-SY5Y cells.

### IRS2 overexpression partially reverses the effects of miR-1277-5p in the cell model of Parkinson’s disease

Lastly, we explored the functional interaction between miR-1277-5p and IRS2 in the cell model of Parkinson’s disease. We transfected IRS2 expression vector to upregulate the IRS2 level in SH-SY5Y cells (Figure 6a). In MPP+ induced cells, miR-1277-5p overexpression could promote cell proliferation and attenuate apoptosis in the cell model of Parkinson’s disease, and the upregulation of IRS2 attenuated these effects (Figure 6b). We further performed ELISA and showed that both the pro-inflammatory cytokines and cellular oxidative stress (ROS and MDA) elicited by MPP+ were suppressed by miR-1277-5p overexpression mimic (Figure 6d), which was accompanied by the increased level of antioxidant enzyme SOD (Figure 6i). The overexpression of IRS2 largely reversed the above effects (Figure 6d-I), Together, these data indicate that IRS2 is a downstream factor mediating the effects of miR-1277-5p in the cell model of Parkinson’s disease.

**Figure 6.** **Upregulating IRS2 reverses the effect of miR-1277-5p overexpression in MPP^+^ induced SH-SY5Y cells**. (a) In the SH-SY5Y cells, compared with the control vector, the transfection of IRS2 expression vector significantly increased protein level of IRS2. (b) CCK-8 proliferation assay in MPP+ induced SH-SY5Y cells with or without miR-1277-5p mimic and IRS2 overexpression. (c) Flow-cytometry based apoptosis detection in MPP+ induced SH-SY5Y cells with or without miR-1277-5p mimic and IRS2 overexpression. (d-i) ELISA was performed to detect (d) TNF-α, (e) IL-1β, (f) IL-6, (g) ROS level, (h) MDA and (i) SOD in MPP+ induced SH-SY5Y cells with or without miR-1277-5p mimic and IRS2 overexpression. Data are the summary of 3 independent experiments. *p < 0.05, **p < 0.01, ***p < 0.001.

## Discussion

Previous studies have showed that non-coding RNAs plays important roles in neurological diseases [23]. Recently many lncRNAs have been implicated in regulation of the pathogenesis of Parkinson’s disease [24]. LncRNA SNHG10 lncRNA was previously reported to contribute to colorectal cancer cells progression by targeting miR-3690 [25]. However, the potential roles of SNHG10 in Parkinson’s disease remain unknown. The current study demonstrated that SNHG10 regulates cellular damage in the cell model of Parkinson’s disease through the miR-1277-5p/IRS2 axis, which may provide novel insights into the mechanisms underlying Parkinson’s disease progression.

Parkinson’s disease is one of the most prevalent neurodegenerative disorder, which is characterized by the progressive loss of dopaminergic neurons and the presence of intraneuronal α-synuclein inclusions [26]. The accumulation of α-synuclein promotes neuroinflammation in Parkinson’s disease [27] and the neuroinflammation contributes to the progression of Parkinson’s disease [28]. Emerging evidence indicate that the dysregulation of lncRNAs are implicated in dopaminergic neuron loss and α-synuclein aggregation [29]. LncRNA NEAT1 (nuclear enriched abundant transcript 1) sponges microRNA-124-3p to upregulate phosphodiesterase 4B (PDE4B), which accelerates the progression of Parkinson’s disease [30]. In addition, lncRNA SOX2-OT (SRY-box transcription factor 2 overlapping transcript) controls cellular damages in the cell model of Parkinson’s disease by regulating the microRNA-942-5p/nuclear apoptosis-inducing factor 1 axis [31]. These studies highlighted the important interactions between lncRNAs and microRNAs in regulating the progression of Parkinson’s disease.

Our data add novel evidence of the implication of lncRNA SNHG10 in cell model of Parkinson’s disease. The functional roles of lncRNA SNHG10 was mainly reported in the digestive tract and respiratory system tumors [32–34]. Here, in the cell model of Parkinson’s disease induced by MPP+, we showed that the expression level of SNHG10 was significantly increased, which was accompanied by the decreased expression of miR-1277-5p. The functional interactions between SNHG10 and miR-1277-5p were validated by functional assays. Importantly, silencing SNHG10 or overexpressing miR-1277-5p could attenuate the inflammatory and oxidative stresses induced by MPP+. Since neuroinflammation is a major factor promoting the progression of Parkinson’s disease [28], these data indicate modulating the expression of SNHG10 and miR-1277-5p could potentially ameliorate the neuroinflammatory condition in Parkinson’s disease, which is needed to be further investigated in the animal model of Parkinson’s disease.

The axis of lncRNA-miRNA-mRNA plays diverse roles in a wide spectrum of diseases [35–37]. In the current study, we demonstrated that the interaction between SNHG10 and miR-1277-5p regulate the expression of downstream target gene IRS2. The functional assays further corroborated that IRS2 acts as a downstream effector mediating the anti-inflammatory and antioxidant effects of silencing SNHG10 or overexpressing miR-1277-5p. Interestingly, a previous study has shown that IRS2 modulates mitochondrial dysfunction and oxidative stress in a mouse model of Huntington disease [38]. Furthermore, dysregulation of IRS2 plays an important inflammatory role in pulmonary vascular remodeling under hypoxic conditions [39]. The above evidence pinpoints the emerging role of IRS2 in regulating inflammatory and oxidative stresses in disease settings. Future studies could focus on the roles of IRS2 and its mechanism in the regulation of inflammatory and oxidative stresses of Parkinson’s disease.

## Conclusion

In summary, our study demonstrated the functional role of SNHG10-miR-1277-5p-IRS2 axis in the regulation of inflammatory and oxidative stresses in the cell model of Parkinson’s disease. These data suggest that modulating the expression of SNHG10 and miR-1277-5p could potentially ameliorate the neuroinflammatory condition in Parkinson’s disease, which requires future validation in animal model of Parkinson’s disease.

## Highlights

- SNHG10 targets miR-1277-5p in the Parkinson’s disease model of MPP+ induced SH-SY5Y cells.
- SNHG10 regulates IRS2 expression by sponging miR-1277-5p in SH-SY5Y cells.
- Knockdown of SNHG10 mitigates MPP+ induced damage via the miR-1277-5p/IRS2 axis.
